The article "Role and Mechanism of Epithelial-Mesenchymal Transition Mediated by Inflammatory Stress-Induced TGF-β1 in Promoting Arteriovenous Fistula Stenosis" was retracted in 2023. Reasons: unreliable results or conclusions; concerns about the data; concerns about the peer review; concerns about the citations.

# Role and Mechanism of Epithelial-Mesenchymal Transition Mediated by Inflammatory Stress-Induced TGF-*β*1 in Promoting Arteriovenous Fistula Stenosis

**DOI:** 10.1155/2022/9454843

**Published:** 2022-07-06

**Authors:** Qingqing Duan, Xiaogang Shen, Dongyuan He, Yuankai Xu, Zhigui Zheng, Zhibo Zheng, Xinxin Jiang, Min Ren, Lili Chen, Ting Zhang, Yunan Lu, Luxi Ye, Xiaohui Xie

**Affiliations:** ^1^Nephrology Department, Zhejiang Hospital, Hangzhou 310012, China; ^2^Nephrology Department, Zhejiang Provincial Peoples' Hospital, Hangzhou 310014, China; ^3^The Department of Obstetrics and Gynecology, Zhejiang Hospital, Hangzhou 310012, China

## Abstract

**Objective:**

To explore the role and mechanism of epithelial-mesenchymal transition (EMT) mediated by inflammatory stress-induced TGF-*β*1 in promoting arteriovenous fistula stenosis.

**Methods:**

The inflammatory cells HK-2 were cultured by adding TGF-*β*1. The optimal stimulation time was determined after TGF-*β*1 was added. HK-2 cells were divided into two groups, DMEM/F12 medium was added to one group (the control group), and the other group was treated with TGF-*β*1 (10 ng/ml) in serum-free DMEM/F12 medium to stimulate cell differentiation to mesenchymal.

**Results:**

TGF-*β*1 was stably expressed after being transfected into EMT. The expression of TGF-*β*1 in the experimental group was higher than that in the control group (*P* < 0.05) 7 days after transfection. Western blot showed that TGF-*β*1 protein expression was higher in the experimental group 7 days after transfection, and no TGF-*β*1 protein expression was detected in the control group. The smooth muscle cells showed *α*-SMA expression in the control group, but no cells with expression of SMA and CD31/vWF were found at the same time; *α*-SMA expression was shown in smooth muscle cells and proliferative myofibroblasts, but no cells with expressions of SMA and CD31/vWF were found at the same time. The observation group showed that the expression of *α*-SMA was detected in smooth muscle cells and proliferative myofibroblasts, CD31/vWF was also expressed in endothelial cells, and *α*-SMA and vWF were also observed in endothelial cells, but no CD31 expression was found.

**Conclusion:**

The inflammatory stress-induced TGF-*β*1 could act on epithelial-mesenchymal transition and promote the degree of arteriovenous fistula stenosis.

## 1. Introduction

Arteriovenous fistula is a commonly used treatment for patients with clinical uremia who often have complications such as arteriovenous fistula stenosis. Studies have shown that myofibroblasts are associated with fistula stenosis in patients. Myofibroblasts are associated with the epithelial-mesenchymal transition (EMT), which is mediated by transforming growth factor *β*1 (TGF-*β*1) [1]. TGF-1 has regulating effects on cell growth, transition, and migration. EMT is the transformation of epithelial cells into mesenchymal cells under certain conditions. It is the binding of transcription factors to target genes caused by some signaling pathways activated by growth factors in EMT, so there is a certain relationship between them [2]. Studies have found that EMT is the main mechanism of fibrosis in the kidney, lungs, and heart, so it can be used as a new target for the treatment of fibrosis diseases [3]. However, the mechanism of TGF-*β*1 mediated EMT and arteriovenous fistula stenosis is still unclear in clinical practice. This study intends to observe the expression of target genes and the regulation of arteriovenous fistula stenosis through inflammatory stress response, and the specific studies are as follows.

The article "Role and Mechanism of Epithelial-Mesenchymal Transition Mediated by Inflammatory Stress-Induced TGF-β1 in Promoting Arteriovenous Fistula Stenosis" was retracted in 2023. Reasons: unreliable results or conclusions; concerns about the data; concerns about the peer review; concerns about the citations.

## 2. Materials and Methods

### 2.1. Instrument and Reagent

Renal tubular epithelial cell HK-2 (Zhongda Hospital Affiliated to Southeast University); EGFP-TGF-*β*1 gene (Shanghai Jikai Genetic Chemistry Technology Co., Ltd.); TRIzol extractant (Shanghai Enzyme-Linked Biotechnology Co., Ltd.); Lipofectamine 2000, Western Blot kit, DEME culture medium, CO_2_ culture medium, and fluorescein secondary antibody (Seymour Fisher); anhydrous ethanol and PBS (Zhejiang Lianshuo Biotechnology Co., Ltd.); *α*-SMA and CD31 antibodies (Shanghai Jining Industrial Co., Ltd.); citrate (Suzhou Tenghao Huagong Technology Co., Ltd.); xylene (Chengdu Puxin Chemical Co., Ltd.); DAPI (GLPBIO, USA). real-time PCR instrument, nucleic acid protein tester, and gel electrophoresis apparatus (Seymour Fisher); embedding machine (Xiaogan Yaguan Medical Electronic Technology Co., Ltd.); paraffin slicer (Hubei Xiaogan Kuahai Medical Technology Co., Ltd.); fluorescence microscope (Leica, Germany).

### 2.2. Cell Culture and Passage

Hk-2 cells were routinely cultured in DMEM medium containing 10% FBS in an incubator with a saturation concentration of 5% CO_2_ at 37°C. Passage: 0.25% trypsin was used for digestion, 1/4∼1/6 ratio was used for passage, and liquid was changed every 2∼3 days. According to the instructions, walmanin (0.2, 0.4, 0.6, 0.8, 1.0, and 1.2 mol/L) and SB203580 (2.5, 5.0, 10.0, 20.0, 40.0, and 50.0 mol/L) were rendered to determine the optimal stimulation concentration and time. Walmanin with a concentration of 1.0 *μ*mol/L + SB203580 10 *μ*mol/L was finally determined to act on for 48 hours.

### 2.3. Effect of TGF-*β*1

The inflammatory cells HK-2 were taken for trypsinization and agitated well to make full contact with the cells. The cells were cultured by adding different concentration gradients of TGF-*β*1 (0, 1, 5, and 10 ng/ml) for 24 hours to select the optimal concentration. The optimal stimulation time was determined after TGF-*β*1 (10 ng/ml) was added and cultured for different time periods (0, 12, 24, and 48 hours).

The article "Role and Mechanism of Epithelial-Mesenchymal Transition Mediated by Inflammatory Stress-Induced TGF-β1 in Promoting Arteriovenous Fistula Stenosis" was retracted in 2023. Reasons: unreliable results or conclusions; concerns about the data; concerns about the peer review; concerns about the citations.

With the determination of the optimal concentration gradients and optimal stimulation time, HK-2 cells were divided into two groups, DMEM/F12 medium was added to one of them (the control group) and the other group was treated with TGF-*β*1 (10 ng/ml) in serum-free DMEM/F12 medium. Each group was equipped with three polypores and the cells were collected after a 24 h culture. The morphological changes in both groups were observed using an inverted phase contrast microscope.

### 2.4. Extraction of Total RNA

With the 24 h cell culture, the original culture medium was discarded and washed twice with PBS solution. Then, the medium was centrifuged at 1000r/min at room temperature for 3 min, the supernate was discarded, and 0.5 ml TRIzol reagent was added and placed at room temperature for 10 min until the cells were completely lysed. Then, 0.1 mL chloroform was added and vigorously mixed for 15 s. The liquid was milky white and was then kept at room temperature for 2 min. The centrifuge was placed at 4°C and centrifuged at 12000 r/min for 10 min. After stratification, the centrifuge was transferred to a new EP tube. Protein and other impurities were not allowed to be inhaled. Isopropyl alcohol was added to the supernate, mixed with the spearhead, kept at room temperature for 10 min, and centrifuged at 12000 r/min, for 10 min at 4°C. It could be seen that the bottom was closed to form an opalescent precipitate, which could be regarded as RNA. The sediment was washed by adding 0.5 ml 75% ethanol into the tube, and the RNA was bounced off the tube wall and fully washed. RNA purity was determined by using standard procedures.

### 2.5. Western Blot

After transfection for 7 days, various cells were collected by cell scraping, total cell protein was extracted, and TGF-*β*1 protein concentration was determined by the BCA method; the samples were quantitatively tested by 10% SDS - ammonium polyacrylamide gel electrophoresis, transferred to the PVDF membrane, sealed with 5% skimmed milk powder for 2 h, added with a 1 : 100 rabbit anti-mouse TGF-*β*1 primary antibody, and left overnight at 4°C. The infrared fluorescence imaging system was used for imaging.

### 2.6. PCR Detection

The cDNA was obtained by reverse transcription with the kit. The PCR reaction conditions were as follows: 1 min at 95°C, 5 s at 95°C, 30 s annealing at 60°C, and 10 min extension at 72°C after 40 cycles. The primer sequences are shown in Table 1.

The article "Role and Mechanism of Epithelial-Mesenchymal Transition Mediated by Inflammatory Stress-Induced TGF-β1 in Promoting Arteriovenous Fistula Stenosis" was retracted in 2023. Reasons: unreliable results or conclusions; concerns about the data; concerns about the peer review; concerns about the citations.

### 2.7. Immunohistochemical Staining

The sections were dewaxed with water and repaired with a citrate antigen at high temperature. The 50% fetal calf serum was sealed at room temperature for 1 h, and the primary antibody CD31/vWF was kept overnight at 4°C; the luciferin secondary antibody was incubated at room temperature for 1 h, washed with PBS buffer solution for 3 times, and sealed with 2.4.5DAPI 6L tablets.

Microvascular count: the number of stained microvessels was searched under a low power microscope (410 times) and counted under 5 high power microscopes (40 × 10 times), and the mean value was taken as the final number of microvessels. If there is a clear separation between the stained cells or cell masses and the surrounding microvessels or tissue structure, it can be considered as numerable microvessels (vessels with lumen diameter being equal to or less than 8 red blood cells and small posterior wall vessels). The percentages of *α*-SMA or CD31/vWF positive to CD31 positive in both groups were calculated, respectively.

### 2.8. Statistical Analysis

The statistical software SPSS22.0 was used for data processing, counting data were represented by “*n* (%),” and tested by the chi-squared test. Measurement data were expressed as *x* ± *s* and tested by “*t*.” *P* < 0.05 indicated that the difference was statistically significant.

## 3. Results

### 3.1. Effect of TGF-*β*1 on Cell Morphology

All cells of the control group were arranged and grown in a pebble-like manner during the culture process, and most of the cells grew adherent to the wall (Figure 1(a)); in the observation group, 24 h after induction, intercellular gaps and tight junctions disappeared; most of the cells were fusiform and fibroid cells appeared (Figure 1(b)).

### 3.2. Comparison of TGF-*β*1 mRNA and Expression of Protein in Both Groups

The PCR results showed that TGF-*β*1 mRNA and protein had been stably transfected into EMT. The expression of TGF-*β*1 mRNA in the experimental group increased gradually and was higher than that in the control group (*P* < 0.05) 7 days after transfection. Western blot showed that TGF-*β*1 protein positive expression was higher in the experimental group, no TGF-*β*1 protein expression was detected in the control group, and the difference between each group was statistically significant (*P* < 0.05), as shown in Table 2 and Figure 2.

### 3.3. Comparison of *α*-SMA and CD31/vWF Expression in Both Groups

The smooth muscle cells showed *α*-SMA expression in the control group, but no cells with expression of SMA and CD31/vWF were found at the same time (Figures 3(a) and 3(b)); *α*-SMA expression was observed in smooth muscle cells and proliferative myofibroblasts, but no cells with expressions of *α*-SMA and CD31/vWF were found at the same time (Figures 3(c) and 3(d)). The observation group showed that the expression of *α*-SMA was detected in smooth muscle cells and proliferative myofibroblasts, CD31/vWF was also expressed in endothelial cells, and *α*-SMA and vWF were also observed in endothelial cells, but no CD31 expression was found (Figures 3(e) and 3(f)).

The article "Role and Mechanism of Epithelial-Mesenchymal Transition Mediated by Inflammatory Stress-Induced TGF-β1 in Promoting Arteriovenous Fistula Stenosis" was retracted in 2023. Reasons: unreliable results or conclusions; concerns about the data; concerns about the peer review; concerns about the citations.

## 4. Discussion

At present, the mechanism of internal fistula vascular stenosis is not obvious in clinical practice, so there is a lack of effective diagnostic methods. Relevant studies have shown that most patients suffer from arteriovenous fistula stenosis due to neointimal hyperplasia, that is, deposition of the extracellular matrix, and formation of microvessels and myofibroblasts [4]. Xiong et al. [5] pointed out that epithelial cells and endothelial cells are very important for disease progression and can effectively participate in wound healing, pulmonary artery hypertension, and atherosclerosis. During EMT, the expression of CD31 and vWF markers was downregulated, and the transfer and diffusion capacity of *α*-SMA was enhanced [6]. Therefore, *α*-SMA and CD31/vWF were used in this study to explore the degree of arteriovenous fistula stenosis.

TGF-*β*1, a polypeptide growth factor, is the initial inducer of EMT, causing the normal intercellular connections to become curved and malleable, thereby causing cells to break away from epithelial tissue. TGF-*β*1, as an inflammatory factor, can effectively act on the immune regulatory process. TGF-*β*1 is released through vascular endothelial cells, and then induces lymphocytes and macrophages to aggregate to the damaged site, thus promoting the synthesis of various inflammatory factors such as fibrocyte proliferation [7]. In addition, the result of Wang et al. [8] showed that the amount of cytokines, chemokines, and other bioactive molecules in the extracellular matrix was changed. TGF-1 is activated by protein spitting and cell membrane protein interaction, and binds to the receptor to produce signals. Inflammatory stress response can activate the static TGF-*β*1, thereby activating the TGF-*β*1-related signal medium expression, and thus regulating the strength of response to EMT [9,10]. The studies of Duan and Derynck [11] and Lin et al. [12] pointed out that SMADS and non-SMADS pathways participated in EMT induction, and exerted regulatory effects on various factors of the extracellular matrix and cell membrane. All cells of the control group were arranged and grown in a pebble-like manner during the culture process, and most of cells grew adherent to the wall; in the observation group, 24 h after induction, intercellular gaps and tight junctions disappeared, and most of the cells were fusiform and fibroid cells appeared, suggesting that TGF-*β*1 induced EMT successfully.

The article "Role and Mechanism of Epithelial-Mesenchymal Transition Mediated by Inflammatory Stress-Induced TGF-β1 in Promoting Arteriovenous Fistula Stenosis" was retracted in 2023. Reasons: unreliable results or conclusions; concerns about the data; concerns about the peer review; concerns about the citations.

The formation of arteriovenous fistula will cause vascular smooth muscle cell proliferation and vessel wall thickening, among which angiotensin-II is one of the key factors. Angiotensin-II can effectively promote the synthesis of TGF-*β*1 and several hypertrophies of vascular smooth muscle cell proliferation, thus causing vascular stenosis [13]. A large number of studies have shown that the cause of arteriovenous fistula stenosis is neointimal hyperplasia [14]. At present, it is believed that the main causes of intimal hyperplasia include inflammation, cell migration, and vascular endothelial cell injury. TGF-*β*1 is biologically active and may be related to neointimal hyperplasia and other pathogenesis. Some studies indicated that TGF-*β*1 was highly expressed in the proliferative veins, and the degree of endometrial hyperplasia significantly increased upon TGF-*β*1 injection [15]. Other studies indicated that the duration of arteriovenous fistula in patients with a high expression of TGF-*β*1 on dialysis is usually significantly shortened in patients with low expression [16], which suggests that TGF-*β*1 may have a significant correlation with the occurrence and development of intimal hyperplasia. In this study, TGF-*β*1 overexpression was speculated to be a major local feature of vascular injury in patients. The PCR results showed that the expression degree of TGF-*β*1 mRNA increased gradually and was higher than that in the control group 7 days after transfection (*P* < 0.05); western blot showed that the TGF-*β*1 protein positive expression was higher in the experimental group, and no TGF-*β*1 protein expression was detected in the control group (*P* < 0.05), which suggested that TGF-*β*1 mRNA and protein were stably transfected into EMT and were expressed for a long time.

Kainum et al. [17] found in cell tracking that EMT appeared in the fibrosis of the kidney, liver, and other organs in patients. The smooth muscle cells showed *α*-SMA expression in the control group, but no cells with expression of SMA and CD31/vWF were found at the same time; *α*-SMA expression was observed in smooth muscle cells and proliferative myofibroblasts, but no cells with expressions of *α*-SMA and CD31/vWF were found at the same time. The observation group showed that the expression of *α*-SMA was detected in smooth muscle cells and proliferative myofibroblasts, CD31/vWF was also expressed in endothelial cells, and *α*-SMA and vWF were also observed in endothelial cells, but no CD31 expression was found. It suggests that TGF-*β*1-mediated EMT is of great significance in the process of arteriovenous fistula stenosis. Weng et al. [18] found that EMT can effectively participate in the process of renal fibrosis; in addition, Yeh et al. [19] pointed out that EMT would lead to loss of the endothelial layer and accumulation of fibroblasts in the intima of blood vessels in late fibrosis. Yan et al. [20] found that patients diagnosed with uremia and undergoing over 2-year hemodialysis also had neointimal hyperplasia, suggesting that regular treatment could also lead to arteriovenous fistula stenosis. This study verified that EMT mediated by TGF-*β*1 high expression was closely related to patients with arteriovenous fistula stenosis, providing an idea for clinical study. The sample size of this study is small, which needs to be increased for further study; moreover, the studies on the correlation between endometrial hyperplasia and TGF-*β*1 expression and the relationship between the TGF-*β*1 signaling pathway and arteriovenous stenosis can be increased in the future. In addition, further studies will be carried out on the protection of patients' arteriovenous vessels.

The article "Role and Mechanism of Epithelial-Mesenchymal Transition Mediated by Inflammatory Stress-Induced TGF-β1 in Promoting Arteriovenous Fistula Stenosis" was retracted in 2023. Reasons: unreliable results or conclusions; concerns about the data; concerns about the peer review; concerns about the citations.

In conclusion, arteriovenous fistula stenosis is a recurrent complication of patients in clinical practice, and TGF-*β*1 mediated EMT can effectively promote arteriovenous fistula stenosis. Meanwhile, with the continuous improvement of the safety of gene transfer technology, this study suggests that some transferred genes can effectively act on local blood vessels to inhibit nitric oxide synthetase, vascular endothelial growth factor, etc., thereby inhibiting neointimal hyperplasia and preventing neointimal hyperplasia of internal fistula.

## Figures and Tables

**Figure 1:** Effect of TGF-*β*1 on cell morphology.

**Figure 2:** Expression of TGF-*β*1 protein in cells 7 days after transfection.

**Figure 3:** Comparison of *α*-SMA and CD31/vWF expressions in both Groups. (a) The expression of fluorescein antibody SMA in smooth muscle cells of SMA and CD32/vWF was not found; (b) the expression of fluorescein antibody SMA in smooth muscle cells; (c) the expression of cytofluorescein antibody SMA in proliferative myofibroblasts; (d) the expression of fluorescein antibody SMA in smooth muscle cells and proliferative myofibroblasts; (e) the expression of fluorescein antibody CD31/vWF in endothelial cells; (f) the expression of fluorescein antibody -SMA and vWF in endothelial cells.

**Table 1:** PCR primer sequences.

Gene	Upstream primer	Downstream primer	Length of product (bp)
TGF-*β*1	5'-CTGCTCCTAGAGCCTCCTGA-3'	5'-GCCCTAATTTTCGGGCATCCT-3'	112
GAPDH	5'-ACAACTTTGGCATCGTGGA-3'	5'-CTTCTGAGTGGCAGTGATGG-3'	62

The article "Role and Mechanism of Epithelial-Mesenchymal Transition Mediated by Inflammatory Stress-Induced TGF-β1 in Promoting Arteriovenous Fistula Stenosis" was retracted in 2023. Reasons: unreliable results or conclusions; concerns about the data; concerns about the peer review; concerns about the citations.

**Table 2:** Relative expression of TGF-*β*1 mRNA in cells 7 days after transfection ($\bar{x}\pm s$).

Group	Cases	The 7^th^ day	
		mRNA	Protein expression
Control group	15	0.287 ± 0.116	—
Experimental group	15	0.685 ± 0.127	0.209 ± 0.007
*t*	8.962	—	—
*P*	0.001	—	—

## Data Availability

The data used to support the findings of this study are available from the corresponding author upon request.
